This article has been retracted.

# Investigation of the Effect of Oral Implant Surgery on Clinical Treatment and Oral Function of Patients with Dentition Loss

**DOI:** 10.1155/2022/1698842

**Published:** 2022-09-21

**Authors:** Bei Men, Shu Jiang, Yongjun Li

**Affiliations:** Dazhong Stomatological Hospital, Wuhan 430000, China

## Abstract

In order to investigate the effect of oral implant surgery on clinical treatment and oral function of patients with dentition loss, a total of 118 patients with dentition loss in the Department of Stomatology of our hospital from January 2019 to January 2022 are retrospectively analyzed. They are randomly divided into the conventional group and the implant group. The conventional group is treated with conventional dentition restoration, and the implant group is treated with oral implant restoration. The repair efficiency of the two groups is compared. The swallowing function of the 2 groups is assessed by Standard Swallowing Assessment (SSA) table before and after treatment. Self-rating depression scale (SDS) and self-rating anxiety scale (SAS) are used to compare the negative emotions of the two groups before and after treatment. Experimental results show that the total effective rate of the implant group is significantly higher than that of the conventional group, but no invalid cases occurred in the two groups after treatment.

## 1. Introduction

Edentulous is a dental disease with a high incidence in the elderly population, which refers to the total loss of maxillary or mandibular teeth due to various reasons. According to research data, the incidence of edentulous in the elderly population is as high as 10.51% [1]. Dentition loss has a great impact on patients, which will not only greatly reduce the masticatory function of patients but also affect the pronunciation function and also reduce the beauty of patients' faces, bringing serious psychological disorders to patients, so timely treatment is essential [2]. The main clinical treatment for dentition loss is the use of denture-assisted fixation therapy. Although it is effective in the short term, long-term use will lead to the loosening or fracture of a denture and other problems, causing a great impact on the physical and mental health of patients [3].

With the development of science and technology, oral implant repair technology has been widely used as a new treatment method. According to the oral conditions of different patients, the technology can select different materials to implant the root, which can not only ensure the completion of dentition missing but also ensure the stability of the implant and ensure a satisfactory effect for patients [4]. Therefore, in this study, a controlled experiment is set up to further compare the differences between oral implants and conventional prostheses, and to explore the clinical efficacy and oral function improvement effect of total prostheses for patients with dentition loss.

The rest of this paper is organized as follows: Section 2 discusses related work.  Section 3 is the treatment methods and self-rating anxiety scale. The comparisons between negative emotions and treatment satisfaction are discussed in Section 4.  Section 5 concludes the paper with a summary.

## 2. Related Work

Dentition loss had a serious impact on patients' masticatory and articulation functions and also damaged patients' physiological function and mental health, which was a kind of dental multiple oral diseases [5, 6]. Therefore, physicians should pay attention to the degree, number, location, and other factors of patients' defects in clinical treatment. As the repair effect of conventional dentures was only average, and there was still an obvious gap between a conventional denture and natural teeth, various functions of patients were difficult to achieve the expected recovery effect, thus affecting the esthetic degree [7]. With the development of science and technology, implant prosthodontic technology has been constantly improved and has been widely used in large medical institutions, which could be more closely combined with dental bone by using materials with high fitness for the human body as a dental base [8].

The discomfort in daily use was lower, and it could make the teeth look no different from those of healthy people, so the clinical efficiency was higher [9]. Because of the higher stability, the oral implant could better assist the swallowing function [10]. It could improve patients' sense of self-efficacy, thus reducing depression, anxiety, and other emotions [11, 12]. Oral implants could be repaired by implanting highly suitable materials in the missing teeth, which could, on the one hand, cover the exposed dental nerve and on the other hand improved the occlusal ability, thus enhancing the chewing function of patients [13]. Since the materials used in oral implants were highly adaptable to human bones, the postoperative rejection reaction was relatively small, and the implant could be closely combined with the gingiva, thus improving the retention function and pronunciation ability [14]. The long-term efficacy of the two groups of patients would be followed up and observed, and the occurrence of adverse reactions would be counted to make the study results more rigorous and reliable [15, 16].

## 3. Treatment Methods and Self-Rating Anxiety Scale

### 3.1. General Information

A total of 118 patients with dentition loss in the Department of Stomatology of our hospital from January 2019 to January 2022 are retrospectively analyzed. The patients are numbered sequentially and put into Excel, singular patients are included in the routine group, and even patients are included in the implant group, with 59 patients in each group. In the conventional group, there are 27 female patients and 32 male patients, aged from 61 to 74 years, with an average of (66.35 ± 6.36) years, with a course of 1 to 3 years, with an average of (2.12 ± 0.53) years. In the implant group, there are 25 female patients and 34 male patients, aged from 62 to 74 years, with an average of (66.72 ± 6.21) years, and the disease course ranged from 1 to 4 years, with an average of (2.32 ± 0.59) years. There is no significant difference in general data between the two groups (*P* > 0.05), which is comparable.

All patients enrolled in the study signed informed consent are as follows: (1) The examination method used in this study is safe, and the examination measures adopted are safe methods that have been used in clinical practice. (2) If you have any discomfort during treatment, please inform your competent doctor in time so as to decide the next treatment plan. (3) The whole treatment and observation period is 3 months, please inform the doctor of your condition change in time. During the treatment, do not use any other drugs or other treatment methods for the disease. If you use them, please inform the doctor. (4) During the study, the original data (including the test sheet) belongs to the research group, but we will protect your privacy. (5) Your participation is entirely voluntary. You have the right to choose not to participate in this study or to withdraw at any time without affecting the normal treatment of your disease. However, I hope to complete this study as far as possible without any special reasons. In any case, please inform your physician.

Inclusion criteria were as follows: (1) Meet the clinical diagnostic criteria for dentition loss. (2) All signed informed consent. (3) No mental diseases. (4) Complete clinical data.

Exclusion criteria were as follows: (1) Oral infection. (2) Communication barriers and inability to cooperate with research. (3) If contact is lost during observation, periodic review is performed. (4) Patients with treatment contraindications.  Table 1 is a general information comparison. It is clearly evident from Table 1 that the degree of education in primary and below of the regular group is almost the same as that in the planting group.

### 3.2. Our Methods

Figure 1 is the treatment satisfaction rate survey in this study.

The conventional group receives conventional denture treatment, and the specific operations are as follows: For patients with gingival disinfection first, and then to local anesthesia, the occlusion is observed and recorded, pull out some residual teeth, determine the distribution of the teeth in the mouth, add braces to do a good job of the artificial tooth row, made for patients in accordance with the oral environment of the denture, and after soaking in 10% mercuric chloride solution, wear in patients with the oral cavity. Attention should be paid to short-term fasting of hard food within 30 days to ensure the stability of the denture and ensure the curative effect.

The implant group receives oral implant repair treatment, which is divided into two steps. The first step is as follows: Using local anesthetic drugs, first look inside the oral environment, locate missing teeth, an alveolar ridge on the appropriate position of about 1 cm incision, cut to ensure that the hard palate sticky periosteum and bone surface exposure, positioning the location of the nest, planting more widen to nest at just the right size, with appropriate concentration of salt water to clean, then implant and fixed in full, and rinse again with the salt water of appropriate concentration. 3 to 6 months after the above treatment is completed, the patient's recovery is checked by X-ray, and the implants that meet the requirements will be treated in the second step. The second treatment operation is as follows: local anesthesia, implant the abutment according to the patient's condition, remove the invalid tissue, check the implantation site, and remove the invalid tissue again. The incision position is accurate and the length is appropriate. According to the patient's oral condition, determine the abutment condition, fix the abutment, tighten the bolts with the help of tools and wear the healing cap, and finally suture the wound. After surgery, the patients are asked to return to the clinic regularly and given appropriate antibiotic treatment. Meanwhile, they should pay attention to fasting on hard food and oral hygiene habits in the short term. Three months later, the oral function, mood change, and esthetic degree of patients in the two groups are observed.

Self-rating anxiety scale (SAS) is used to evaluate the degree of psychological anxiety of patients and the changes in the treatment process, and score the patients' anxiety, fear, fear, breathing, and other conditions. The scoring system adopts a 4-level score, and no or little is recorded as 1 point. A small amount of time is 2 points; most of the time, 3 points; most or all of the time is 4 points. A total score below 50 is normal, 50–70 is classified as an anxious state, and over 70 is classified as a severe anxiety state. The higher the score is, the more serious the patient's anxiety mood is.

Self-rating depression scale (SDS) is used to reflect patients' depression and the changes in the treatment process, including 20 items such as depression, easy to cry, and sleep disorder. The scoring system adopts a 4-level scoring system, among which 10 items are positive scoring and the other 10 items are reverse scoring. A score below 53 indicates normal, between 53 and 72 indicates depression, and a score above 72 indicates major depression. The higher the score, the more serious the depression.

If Standard Swallowing Assessment (SSA) is divided into two phases, the first phase may continue in the second stage. The first stage includes giving patients 5 ml of water to swallow and whether in the process of swallowing the water, one needs to record the phenomenon such as cough and hoarseness; if the aforementioned symptoms appear, one is not for the second phase, and if not, more symptoms may be seen in the second stage. In the second stage, patients are given 60 ml of water for swallowing. If the patient has symptoms such as dry air, cough after swallowing, and hoarseness during drinking, it is considered unsafe to swallow. The swallowing function score is 1 and 2 points from no time, and the score ranges from 11 to 25 points. The higher the score, the worse the swallowing function.

The final curative effect is divided into marked effect, effective, cured, and invalid. The missing part of the dentition is completely repaired, and there is no difference in appearance and function compared with healthy teeth, which is regarded as a marked effect. Basic restoration of the missing part of dentition, which is not much different from healthy human teeth in appearance and function, is regarded as effective. Although the missing part of dentition is not completely repaired and there is some discomfort, it does not affect daily life, it is regarded as a cure. If the missing part of the dentition is not repaired effectively and the oral function of speaking and chewing is different from that of normal people, it is regarded as invalid.

The masticatory function, retentive function, esthetic degree, and articulation function of the two groups are determined by the doctor's observation of the patients in all aspects, and the full score of each index is 10 points.

Oral inquiry is used to investigate the nursing satisfaction of patients, satisfaction can be divided into dissatisfied, general, satisfied, and very satisfied. Satisfaction rate = (satisfied + very satisfied)/number of patients × 100%.

### 3.3. Observation Indicators

The observation indicators are as follows:

1. Clinical efficacy is compared.
2. SSA score is used to compare the changes in swallowing function.
3. SAS and SDS scores are used to compare the changes in negative emotions.
4. Masticatory function, retention function, pronunciation function, and esthetic degree are evaluated.
5. The treatment satisfaction rate is compared.

### 3.4. Statistical Processing

All data during the study are collected and sorted out and put into SPSS22.0 for statistical processing. Measurement data are expressed as $\left(\bar{x}\pm s\right)$. Count data are represented by (%), and differences between groups are tested by *x2*. When *P* < 0.05, the difference between data is statistically significant.

## 4. Comparisons of Negative Emotions and Treatment Satisfaction

### 4.1. Comparison of Clinical Efficacy

Table 2 is the clinical curative effect. It is clearly evident from Table 2 that the total effective rate of the implant group is higher than that of the conventional group (*P* < 0.05).

Figure 2 shows the comparison of clinical efficacy. It is clearly evident from Figure 2 that no invalid cases occur in the two groups after treatment.

### 4.2. Comparison of Swallowing Function

Table 3 shows the SSA comparison. It is clearly evident from Table 3 that before treatment, there is no significant difference in SSA (*P* > 0.05).

Figure 3 shows the comparison of swallowing function. It is clearly evident from Figure 3 that the swallowing function is significantly improved after different treatment methods and the improvement degree in the implant group is higher than that in the conventional group (*P* < 0.05).

### 4.3. Comparison of Negative Emotions

Table 4 shows the negative emotion contrast. It is clearly evident from Table 4 that before treatment, there is no significant difference in adverse emotions between the two groups (*P* > 0.05), and the negative emotions are alleviated after treatment, and the degree of depression and anxiety in the implant group are significantly lower than that in the conventional group (*P* < 0.05).

### 4.4. Comparison of Other Functions

Table 5 shows the comparison of other functions. It is clearly evident from Table 5 that before treatment, there are no significant differences in chewing function, retention function, aesthetics, and pronunciation function between the two groups (*P* > 0.05), but after treatment, all functions of the two groups increase, and the implant group performs significantly better than the conventional group in all aspects (*P* < 0.05).

### 4.5. Comparison of Treatment Satisfaction

Table 6 shows the comparison of satisfaction rates. It is clearly evident from Table 6 that the normal satisfaction rate of the regular group is significantly higher than that of the planting group.

Figure 4 shows the comparison of treatment satisfaction. It is clearly evident from Figure 4 that the satisfaction rate of the planting group is significantly higher than that of the conventional group.

## 5. Conclusion

The results of this study show that compared with conventional dentures, the clinical efficacy of the oral implant group is significantly higher than that of the conventional denture group (*P* < 0.05), but there are no invalid cases after surgery in both groups, suggesting that both methods can help with tooth loss. The patient repairs the teeth and gives feedback on the oral function to a certain extent, and the oral implant technology has a high degree of joints due to the use of materials and the body. To sum up, patients using oral implant technology can respond to dentures and oral function, and reduce the negative emotions of patients. Patients can choose different dentures according to their own conditions, but oral implant technology has improved significantly in all aspects. It is superior to dentures, has high clinical value, and is worthy of clinical use.

## Figures and Tables

**Figure 1:** Treatment satisfaction rate survey.

**Figure 2:** Comparison of clinical efficacy.

**Figure 3:** Comparison of swallowing function.

**Figure 4:** Comparison of treatment satisfaction.

**Table 1:** General information comparison.

	Regular group (*n* = 59)	Planting group (*n* = 59)	*t/x2*	*P*
Gender			0.138	0.711
Men	32 (54.24%)	34 (57.63%)		
Woman	27 (45.76%)	25 (42.37%)		

Age	66.35 ± 6.36	66.72 ± 6.21	−0.320	0.750
Course of the disease(year)	2.12 ± 0.53	2.32 ± 0.59	−1.937	0.055
BMI(kg/m^2^)	26.35 ± 4.52	26.98 ± 4.27	−0.778	0.438
The degree of education			0.136	0.713
Primary and below	21 (35.59%)	18 (30.51%)		
Junior to senior high	29 (49.15%)	31 (52.54%)		
University and above	9 (15.25%)	10 (16.95%)		

Spouse situation			0.457	0.499
Y	45 (76.27%)	48 (81.36%)		
N	14 (23.73%)	11 (18.64%)		

**Table 2:** Clinical curative effect.

	Planting group (*n* = 59)	Regular group (*n* = 59)	*x2*	*P*
Excellent	28 (47.46%)	20 (33.90%)		
Effective	23 (38.98%)	22 (37.29%)		
Healing	8 (13.56%)	17 (28.81%)		
Invalid	0 (0.00%)	0 (0.00%)		
Total effective rate	51 (86.44%)	42 (71.19%)	4.111	0.043

**Table 3:** SSA comparison.

	Number	Before the treatment	After the treatment	*t*	*P*
Planting group	59	21.37 ± 1.86	14.33 ± 2.13	19.123	<0.001
Regular group	59	21.42 ± 1.79	17.23 ± 1.82	12.608	<0.001
*t*		−0.149	−7.951		
*P*		0.882	<0.001		

**Table 4:** Negative emotion contrast.

		Regular group (*n* = 59)	Planting group (*n* = 59)	*t*	*P*
Before the treatment	SAS	64.37 ± 8.98	65.25 ± 8.19	−0.847	0.397
	SDS	68.67 ± 6.06	69.17 ± 6.75	−0.645	0.519

After the treatment	SAS	55.27 ± 6.32^*∗*^	42.87 ± 5.91^*∗*^	16.774	<0.001
	SDS	57.25 ± 7.19^*∗*^	49.27 ± 6.93^*∗*^	9.353	<0.001

**Table 5:** Comparison of other functions.

		Planting group (*n* = 59)	Regular group (*n* = 59)	*t*	*P*
Before the treatment	Chewing function	5.31 ± 0.45	5.34 ± 0.42	−0.374	0.709
	Pronunciation function	8.34 ± 0.21	8.31 ± 0.25	0.706	0.482
	Beautiful degree	5.62 ± 1.21	5.73 ± 1.18	−0.500	0.618
	Fixed function	5.53 ± 1.02	5.48 ± 1.06	0.261	0.794

After the treatment	Chewing function	8.42 ± 0.83^*∗*^	7.78 ± 0.72^*∗*^	4.474	<0.001
	Pronunciation function	9.24 ± 0.15^*∗*^	9.03 ± 0.12^*∗*^	8.397	<0.001
	Beautiful degree	8.94 ± 0.56^*∗*^	8.02 ± 0.47^*∗*^	9.666	<0.001
	Fixed function	7.23 ± 1.12^*∗*^	6.64 ± 1.02^*∗*^	2.992	0.003

**Table 6:** Comparison of satisfaction rate.

	Regular group (*n* = 59)	Planting group (*n* = 59)	*x2*	*P*
Dissatisfied	1 (1.69%)	0 (0.00%)		
Normal	15 (25.42%)	7 (11.86%)		
Satisfied	25 (42.37%)	27 (45.76%)		
Very satisfied	18 (30.51%)	25 (42.37%)		
Satisfaction	43 (72.88%)	52 (88.14%)	4.374	0.036

## Data Availability

The simulation experiment data used to support the findings of this study are available from the corresponding author upon request.
